# A Machine Learning-Based Prediction Model for Preterm Birth in Rural India

**DOI:** 10.1155/2021/6665573

**Published:** 2021-06-15

**Authors:** Rakesh Raja, Indrajit Mukherjee, Bikash Kanti Sarkar

**Affiliations:** Department of Computer Science & Engineering, Birla Institute of Technology, Mesra, Ranchi, India

## Abstract

Preterm birth (PTB) in a pregnant woman is the most serious issue in the field of Gynaecology and Obstetrics, especially in rural India. In recent years, various clinical prediction models for PTB have been developed to improve the accuracy of learning models. However, to the best of the authors' knowledge, most of them suffer from selecting the most accurate features from the medical dataset in linear time. The present paper attempts to design a machine learning model named as risk prediction conceptual model (RPCM) for the prediction of PTB. In this paper, a feature selection approach is proposed based on the notion of entropy. The novel approach is used to find the best maternal features (responsible for PTB) from the obstetrical dataset and aims to predict the classifier's accuracy at the highest level. The paper first deals with the review of PTB cases (which is neglected in many developing countries including India). Next, we collect obstetrical data from the Community Health Centre of rural areas (Kamdara, Jharkhand). The suggested approach is then applied on collected data to identify the excellent maternal features (text-based symptoms) present in pregnant women in order to classify all birth cases into term birth and PTB. The machine learning part of the model is implemented using three different classifiers, namely, decision tree (DT), logistic regression (LR), and support vector machine (SVM) for PTB prediction. The performance of the classifiers is measured in terms of accuracy, specificity, and sensitivity. Finally, the SVM classifier generates an accuracy of **90.9%**, which is higher than other learning classifiers used in this study.

## 1. Introduction

Preterm birth (PTB) is a serious public health problem that adversely affects both families and the society [1]. It is a leading cause of neonatal mortality and morbidity across the world and also the second major cause of child deaths under the age of five years [2]. Over the past two decades, PTB has been a significant research study in healthcare domain. Pregnancy and childbirth unlocked the door for medical experts and researchers to explore various effective strategies to reduce preterm birth in women having pregnancy-related complications. These strategies include healthcare services given to all pregnant women to control PTB and any medical interventions aimed to enhance the knowledge of women on early indications of pregnancy complications [3, 4]. The maternal history of a pregnant woman is a key part of the neonatal studies for providing certain clinical treatments to newborn babies regarding their health, disease, care, and outcomes. Newborn babies are very special. They do not have any previous medical background, and their early neonatal path is directly connected to the maternal history of their mothers [5–7]. The healthcare services also incorporate the arrangements of essential social and economic support for women before, during, and after pregnancy including educational, medical, and other training programs that facilitate healthy motherhood.

In general, treatments of diseases (including PTB) are made by the physicians based upon their knowledge (experience). However, on the one hand, manual diagnosis may not be often right as physician's experience varies from expert to expert. On the other hand, manual treatment is a time-consuming job. Further, shortage of medical experts is increasing everyday with population explosion and developing countries like in India, large number of women belong to lower or middle income families. They do not get proper healthcare facilities or awareness regarding health education to know about any complication that arises during pregnancy, especially in rural area. Further, people often are afraid of doctors' prescription since doctors in most cases misguide the patients suggesting unnecessary tests (like double marker test, fetal echocardiography, urine test, and FT4 test which are used to determine any pregnancy complications) which are very expensive. Also, doctor's appointment fees are mostly on higher side. Besides, doctors could sometime diagnose the cases wrongly. After all, preterm delivery is the most critical issue in Gynaecology and Obstetrics and a major health concern for every pregnant woman. It may require several ultrasound sonography (USG) tests in addition to doctor's appointment fee for diagnosing high-risk patients, and these altogether may amount huge expense that may be beyond the income limit of many families. So, designing the computerized system (i.e., e-healthcare system) for birth prediction from past diagnosis data is the essential solution for quick and accurate decision to be taken for any adverse pregnancy outcome in order to save lives and cost.

Notably, a pioneering renovation is taking place in the Obstetrical community due to the advancement in technology and digitization of medical records. Data analytics is one of the most promising tool for research and development in the area of medicine [8–15]. Nowadays, machine learning techniques (e.g., neural networks, support vector machine, logistic regression, and Decision Trees) are playing important role in designing the disease predictive model to address the growing needs of human experts in the medical world [16–20]. However, medical datasets are highly imbalanced, conflicting in nature, and uncertain. So, designing the effective intelligent model for medical datasets is a challenging task. PTB dataset is one such clinical dataset. Numerous predictive models based on standard intelligent methods have been introduced by the researchers for prediction of PTB [21]. However, they usually suffer from several drawbacks like lack of understandability and inefficiency in making quick and correct decision. Further, early detection and diagnosis play important role in controlling such complications. Symptoms (text) based machine intelligent models may play vital role in early detection of such cases. The delay in receiving the clinical judgement for preterm delivery increases the risk of pregnancy complications which in turn increases the risk of prenatal mortality. Due to its direct association with prenatal mortality, neonatal health is also very important in the obstetrical community [7]. According to the UNICEF study released in 2015, 35% of neonatal death is due to PTB. The rate of PTB in rural areas of most developing countries is increasing due to lack of health facilities and insufficient number of healthcare workers.

In light of these considerations, the present study aims to design a novel conceptual model (by employing machine learning techniques) and its implementation for detection of PTB in pregnant women. In fact, the system can be used as a decision support system to assist the medical staff and healthcare workers for predicting premature delivery. More specifically, the present study focuses on novel feature selection (entropy-notion) approach to identify the most important maternal features (text-based symptoms) responsible for preterm delivery and aims to predict the classification accuracy.

The remaining sections of the paper are organized as follows.  Section 2 describes the basic concept of PTB and feature selection.  Section 3 elaborates the related work that has been carried out to predict PTB.  Section 4 describes the methodology of this research. The experimental design and results are presented in Section 5. Finally, Section 6 deals with conclusion and future scopes.

## 2. Background of the Present Research

### 2.1. Preterm Birth (PTB): A Comprehensive Overview

Preterm or premature birth is defined as birth, for any reason, occurring before 37 completed weeks (or less than 259 days) of pregnancy. Every year, about fifteen million babies are born prematurely (before 37 completed weeks of gestation), and this is nearly equal to one-tenth of all babies around the world [22]. According to the WHO reports studied in 2005, 12.9 million births or 9.6% of all births across the world occurred prematurely [23]. The rate of preterm birth, however, significantly varies across the world. Preterm birth reflects the most prominent reason for neonatal morbidity and mortality [24].

#### 2.1.1. Categorization of PTB

PTB can be classified into different categories based on gestational age at birth. The gestational age is defined as the time from the first day of the last menstrual period (LMP) of a woman to birth [21]. The four categories of PTB are as follows:

- *Extreme PTB (under 28 Weeks).* It is the birth that takes place before 28 weeks of pregnancy
- *Very PTB (28 to 32 Weeks).* It is the birth that takes place between 28 and 32 weeks of pregnancy
- *Moderate PTB (32 to 34 Weeks).* It is the birth that takes place between 32 and 34 weeks of pregnancy
- *Late PTB (34 to 37 Weeks).* It is the birth that takes place between 34 and 37 weeks of pregnancy

#### 2.1.2. Medical Terminologies

For the purpose of clarity of the present study, the used terminologies are illustrated in Table 1.

#### 2.1.3. Health Impact of PTB

PTB is the main risk factor for newborn mortality and morbidity. It is a leading cause of neonatal mortality and morbidity across the world and also the second major cause of child deaths under the age of five years [25]. It arises between 5 and 10% of all deliveries and involves 70% of neonatal mortality and up to 75% of neonatal morbidity [26]. Premature infants are more likely to suffer than normal birth and are at higher risk of brain paralysis, sensory impairment, respiratory failure, and so on. More than $13 billon of premature cost for maternity service is anticipated only in the USA [27, 28]. Most survivors of PTB face serious problems, often a lifetime of disability, including learning disabilities, visual, and hearing problems. In fact, babies born premature have more health problems compared with babies born at term birth. Term birth refers to babies that are born at 37 to 40 weeks of gestation. Furthermore, babies born at preterm are reported to be at an elevated risk of long-term health problems [29]. Unfortunately, after many years of research in obstetrics, yet the rate of PTB has not decreased [30]. Birth weight is generally associated with PTB and results in its own categorization. Usually, birth weight is simpler to measure precisely and is a first estimation of gestational age. Obviously, the most challenging issue in Gynaecology and Obstetrics is how to control the preterm delivery in pregnant women.

### 2.2. Feature Selection (FS)

The term feature selection in the machine learning, also known as feature subset selection, refers to the process of selecting a subset of excellent features during construction of the predictive model. The presence of redundant and irrelevant features in any datasets (especially in medical datasets) can reduce the accuracy of the model's prediction and also have the negative impact on the performance of the model. The main goal of any feature selection method is to select the best subset of features by removing redundant and irrelevant features from the datasets in order to reduce the training time and enhance the classifier's predictive performance. In fact, feature selection is typically used as a preprocessing step in data mining. There are three standard approaches of the feature selection algorithm, namely, filter method, wrapper method, and embedded method. For more details about feature selection, one may refer to [31–33].

- *Filter Method*. The filter method measures the relevance of features based on the nature of data. The selection of features is independent of the classifiers used. The filter method is much faster compared with the wrapper method and provides an average accuracy for all the classifiers used. Some of the examples of filter methods are information gain, chi-square test, variance threshold, and so on.
- *Wrapper Method*. The wrapper method finds the best subset of features based on a specific machine learning algorithm that we are trying to fit on a given dataset. The evaluation criteria are simply the predictive power of the particular classifier. The wrapper method has higher performance accuracy compared with the filter method but requires more computational time to find best features for a dataset with high-dimensional features. Some of the examples of wrapper methods are forward selection, backward elimination, genetic algorithms, and so on.
- *Embedded Method*. The embedded method incorporates the advantages of both filter and wrapper methods. In this approach, feature selection is done during the process of model training and is usually unique to particular learning classifiers. This approach basically determines the importance of feature, i.e., which features to accept and which to reject, while making a prediction. The most typical embedded technique is the decision tree algorithm. This method typically falls somewhere between the filter method and wrapper method in terms of time complexity. Some of the examples of embedded methods are lasso regression, ridge regression, elastic net, and so on.

## 3. Related Works

This section focuses mainly on the existing methodologies related to prediction of PTB using machine learning, statistical analysis, and data mining techniques. Some of them are discussed in this section. The study of Mercer et al. [34] was designed to develop a risk-score-based model for predicting PTB. The model can be trained using a multivariate logistic regression technique to explore various risk factors using clinical data available between 23 and 24 weeks' gestation. Goodwin et al. employed the machine learning model to generate 520 predictive rules for PTB with the application of data mining techniques [35]. The study in [36] discussed the deep learning models for predicting preterm delivery using existing electronic medical records (EMRs) of mothers available in healthcare centres.

Weber et al. [37] performed a cohort study to predict spontaneous preterm. The prediction of PTB was performed using numerous classifiers, namely, K-nearest neighbours, lasso regression, and random forests. This study has taken into the consideration of demographic, race-ethnicity, and maternal characteristics. Mailath-Pokorny et al. [38] explored the predictive features for preterm delivery that occurs within 2 days after admission and before 224 days of gestation using the multivariate logistic regression model. The predictive features considered are age of the mother, gestational age during admission, maternal history, vaginal bleeding, cervical length, preterm history, and preterm premature rupture of membranes (PPROM) in their study. Son and Miller presented a prediction model for PTB using cervical length measurement in women with a singleton gestation. To accomplish better predictive performance, they attempted to determine the best cut points of cervical length [39].

Elaveyini et al. [40] explored the major risk factors of preterm birth using artificial neural networks. PTB prediction was based on the feed-forward backpropagation algorithm. Over the past decades, majority of research studies have been done to enhance the accuracy of prediction of PTB [41]. Researchers are continually making their best efforts to analyse and explore the principal risk factors for preterm delivery [42–44]. The present article focuses on the machine learning approaches for prediction of birth cases in rural community.

### 3.1. Shortcomings in the Existing Clinical Models

In recent years, using feature selection approach, a significant number of clinical prediction model have been developed to improve the accuracy of learning models. However, to the best of authors' knowledge, most of them suffer from selecting the most accurate features from the medical dataset in linear time. Hence, there is a scope for improving the performance of machine learning classifiers and reducing learning time.

### 3.2. Novel Contribution

A novel feature selection approach based on the notion of entropy is introduced in this study to address the identified issues of the existing models. The key role of the novel approach is to find the subset of optimal features from the medical dataset in order to improve the prediction's accuracy and ultimately reduce the machine learning time.

## 4. Research Methodology

### 4.1. Objective

The finding of this research study can be utilized to fulfill the three following main objectives:

- A machine learning-based risk prediction conceptual model (RPCM) for PTB can be introduced with the help of novel feature selection approach using entropy-notion to predict the birth cases (TB and PTB) from the obstetrical records.
- The suggested approach is used to identify the excellent (text-based symptoms) features responsible for PTB. Furthermore, medical experts' (physicians and obstetricians) opinions are also considered through review of medical records of patients and survey analysis. The model can be extended to select the regions for pregnancy consultation.
- The predictive model can be beneficial for rural India to identify the important maternal features in order to predict the possibility of PTB in the gestation of women. This information can support rural medical staff for taking effective decisions for adverse pregnancy outcome—that aim to reduce the diagnosis cost.

### 4.2. The Proposed Feature Selection Approach Based on the Notion of Entropy

According to the study in [45], attributes having strong correlation cannot be the part of feature subset. Besides, more the attributes are independent among themselves and more information gain they will have which would eventually give better outcomes over unseen data. The present research focuses on medical (obstetrical) datasets which are more sensitive in nature, so feature selection approach is more effective for such datasets. In light of this point, a feature selection (entropy-notion) approach is presented here to extract the most relevant features from obstetrical (term-preterm) dataset. These features are utilized to classify all birth cases into term birth and PTB. A conceptual model of the proposed approach is shown in Figure 1.

The proposed approach is stated as follows:

- Suppose that *D* is a medical dataset having *n* attributes, say *A*_*i*_ for *i* = 1, 2, 3,…, *n*.
- Let *F*_0_ denote a set of features in the original dataset *D*.
- Initially, *F*_0_ = {*A*_1_, *A*_2_, *A*_3_,…, *A*_*n*_}.
- Since *D* is divided into three distinct subsets as *D*_1_, *D*_2_, and *D*_3_, so after applying the proposed approach, we get three feature subsets, namely, *F*_1_, *F*_2_, and *F*_3_ from these data subsets.
- *F* is considered as a resultant feature set derived from *F*_1_, *F*_2_, and *F*_3_. Initially, *F*_*k*_ = *F*_0_ for *k* = 1, 2, 3.
- Let *P* be a classification problem described by a set of *n* attributes, say *A*_*i*_ for *i* = 1, 2, 3,…, *n* and also consider that *F* represents the set of features derived from the original dataset.
- Initialize, *F* = *F*_0_ = {*A*_1_, *A*_2_, *A*_3_,…, *A*_*n*_}.
- for each data subset *D*_*i*_ ∈ *D*; where *i* = 1, 2, 3
- do
-  for each attribute *A*_*i*_ ∈ *F*_0_
-  do
-   Calculate Gain (*S*, *A*_*i*_)//information gain for *A*_*i*_
-   Using formula stated below,
-    Gain(*S*, *A*_*i*_)=Entropy(*S*) − Σ_*v*_*j*_∈*A*_*i*__(|*S*_*v*_*j*__|/|*s*|)Entropy(*S*_*v*_*j*__), where *v*_*j*_ denotes values of attribute *A*_*i*_ and *Entropy*(*S*)= Σ*p*_*m*_log_2_*p*_*m*_, where *S* represents the number of instances in *P* and *p*_*m*_ is the nonzero probability of *s*_*m*_ instances (out of *S*) belonging to class *m*, out of *c* classes.
-  end for
-   Compute *r*=(*Max*_*Gain*(*S*, *A*_*i*_) −  *Min*_*Gain*(*S*, *A*_*i*_)/*n*), where *i* = 1, 2, 3,…, *n*.
-   //Here, *r* is considered as a threshold value for selecting features
-   for each attribute *Ai* ∈ *F*_0_
-   do
-    if *Gain*(*S*, *A*_*i*_) < *r*
-    then
-    update *F*_*k*_ = *F*_*k*_─{A_*i*_}//removing *A*_*i*_ from *F*_*k*_
-   end if
-  end for
- end for
- *F* = *F*_1_ U *F*_2_ U *F*_3_//including all attributes of *F*_1_, *F*_2_, and *F*_3_.

*Note*. The proposed feature selection approach in this study is a form of the filter method and is implemented in Java-1.4.

*Time Complexity*. The algorithm is simple and easy to understand. The running time of an algorithm is *O*(*n*), where *n* is the number of attributes in the dataset.

### 4.3. The Proposed Framework: Risk Prediction Conceptual Model (RPCM)

Based on novel feature selection (entropy-notion) approach and several studies in [46–49], RPCM is carefully designed to predict the risk of PTB in pregnant women. The workflow of the framework consisting of three stages (Stage-I, Stage-II, and Stage-III) is depicted in Figure 2, and then its each component is detailed.

#### 4.3.1. Key Components of the Proposed Model

The proposed model consists of some key components, namely, healthcare centre, patient survey, maternal and neonatal records, data preprocessing, machine learning, and birth outcome. Each of these is discussed as follows:

- *Healthcare Centre*. A healthcare centre is a part of a network of hospitals employed by a group of general physicians, nurses, and healthcare professionals that provide healthcare facilities to people in a certain area. In addition to standard medical treatments, one of the main goals of the primary healthcare centre is maternal care during pregnancy especially in rural India. This is because people from rural India avoid contacting healthcare professionals and practitioners for pregnancy care which increases the cases of maternal and neonatal deaths.
- *Patient Survey*. A comprehensive care to mother and child is primarily concerned to all healthcare systems in India. The term survey describes any study that consists of requesting people to respond queries. This entails researcher-developed questionnaires and personal interviews with pregnant women during their antenatal care visits.
- *Maternal and Neonatal Records*. Maternal and neonatal records play a vital role in deciding the way healthcare services are provided, accessed, and affected by health outcomes. It stores the statistical reports describing the use of prenatal services, maternal risk factors, and birth outcomes for all patients residing in rural area. PTB is one of the most frequent complication of pregnancy. It occurs due to several medical reasons and is affected by some of the important maternal features based on human experts (experience) and several research studies [50–53]. These maternal features are critical in nature to predict cases of PTB. The total number of birth instances is taken from the obstetrical data.
- *Data Discretization*. A technique of converting continuous values of attribute into a finite set of intervals and associating a new discrete value with each interval is known as data discretization. Since any classifiers prefer to handle discrete values rather than continuous values for the learning process, data discretization plays a crucial role in the process of machine learning. The study in [54] suggests that data discretization improves the quality of discovered knowledge, and it is based on the concept of information theory.
- *Feature Selection*. One of the core concepts in machine learning is the feature selection. Feature selection is the process of selecting those features from the input datasets which highly impact the performance of the predictive model. The present study focuses on feature selection approach based on entropy notion as already discussed in Section 4.2.
- *Data Preprocessing*. The tabular dataset collected from obstetrical data is preprocessed and converted into a normalized form with the help of MIL discretizer [55, 56].
- *Machine Learning (ML)*. The present study focuses on applying machine learning algorithms [46, 49] for PTB prediction. ML is a method of data analysis that automates analytical model building. Classification is one of the most popular approaches for applying ML methods (e.g., DT, LR, and SVM). These techniques are used to in medical domain for classification, prediction, and diagnosis purposes.
- *Birth Outcome*. This component is very crucial in preventing preterm delivery in pregnant women during antenatal care clinics. The predicted birth outcome can also be used to properly analyse the key maternal features responsible for PTB.

### 4.4. Details of Stage-I

The main role of the first stage of framework is to collect obstetrical data from the Community Healthcare Centre, and it is detailed in this section.

#### 4.4.1. Study Design

The study was conducted in the Community Health Centre, Kamdara (Gumla), situated in rural area of Jharkhand, during a period from July 2018 to September 2020. The hospital provides obstetric and gynaecological services to all categories of women, whether registered for antenatal care or referred. The approval for the study was taken from the Institutional Ethics Committee.

*Selection Criteria*. The selection of patients (women) depends on the following inclusion-exclusion criteria:

Inclusion criteria include the following:
  - Women registered for ANC and having birth at the Community Health Centre
  - Women having birth occurring at the gestational age of 28 weeks or more
  - Women who delivered a live birth
Exclusion criteria include the following:
  - Women having still birth
  - Women having birth of twins
  - Women referred to other hospitals

#### 4.4.2. Data Collection

The basic step of Stage-I is to collect data based on patient survey and maternal records available in the obstetrics department. Initially, 1800 records were collected during a research period. Then, 1300 records were selected for further study based upon inclusion-exclusion criteria. The collected records include all instances of term birth and PTB. A manual analysis is performed to select all maternal features which are involved during pregnancy (based on medical experts' opinion and several research studies) [51, 52, 57, 58]. The description of the obstetrical dataset (original) after data collection is summarized in Table 2.

Initially, all instances are in a raw-form which are compiled into a tabular-form using MS Excel program. As a result, a tabular (term-preterm) dataset is prepared for the research purpose. The tabular (term-preterm) dataset used in this work is a binary class dataset.

The feature values in this dataset are of the form-string, integer, and continuous. The tabular (term-preterm) dataset consists of 1300 instances, composed of thirty-six different features which are taken into consideration before, during, and after pregnancy. These features are listed in Table 3. The questionnaire used for data entry during patient survey was mainly focused on their background details, medical history, previous pregnancy details, current pregnancy details, baby details, and medical disorders in current pregnancy.

### 4.5. Description of Stage-II

The collected data from tabular (term-preterm) dataset are preprocessed at the second stage of the framework. This stage deals with two main operations, namely, data discretization and feature selection.

#### 4.5.1. Data Discretization

During data preprocessing, tabular (term-preterm) dataset is converted into a normalized form with the help of data discretization process. This gives a discretized (term-preterm) dataset. This dataset is utilized to select most accurate features by applying suggested feature selection approach based on the notion of entropy. The initial statistics of discretized (term-preterm) dataset is shown in Table 4.

In reality, attributes of any medical dataset may contain mixture of string, continuous, outliers, and missing data. Many classifiers cannot handle continuous attributes but each of them can operate on discretized attributes [55]. Besides, performance of classifiers can be significantly improved by replacing continuous attributes with its discretized values. Depending upon the amount of missing data and the criticality of the feature in which the data is missing, it may impact the accuracy of prediction. In this study, the missing value in any feature is replaced with the mean value of that feature, and minimum information loss (MIL) data discretizer [12, 54, 59] is employed here for data processing, which make data compatible with the machine learning algorithm.

#### 4.5.2. Feature Selection

After that, the proposed feature selection approach is taken into consideration to select the most probable features (responsible for PTB) from the discretized (term-preterm) dataset. As a result, seventeen different features are selected from this dataset. These maternal features (listed in Table 5) are also considered as major risk factors for PTB as suggested by medical experts and several research studies. Then, a final birth (term-preterm) dataset, consisting of these selected features, is prepared for the last stage of framework. The birth dataset also contains 1300 instances of term birth and PTB.

### 4.6. Description of Stage-III

Finally, a machine learning-based prediction model for PTB is built at this stage. This section describes the actual construction of the suggested system.

#### 4.6.1. Machine Learning PTB Model

The aim of this research is to find a suitable classifier which can predict the PTB with more accuracy. The three classifiers, namely, decision tree (DT), logistic regression (LR), and support vector machine (SVM) are used in this analysis. The method of selecting classifier in this study is illustrated in Figure 3. Model fitting was carried out by dividing the input dataset into training dataset and test dataset at a ratio of 70% and 30%, respectively. The training set is used in learning phase and test set is used in prediction phase, to determine the best model. Researchers may find ample information about several machine learning classifiers from the articles [60–63].

#### 4.6.2. Evaluation of Machine Learning Classifiers

The empirical measures can be extracted from the confusion matrix in order to evaluate the performance of the learning classifier [64]. A confusion matrix shows the accuracy of the solution to a classification problem.  Table 6 depicts the confusion matrix, which summarizes the number of instances predicted correctly or incorrectly by a classification model.

Furthermore, the other parameters used to measure the classifier's performance are correct classification rate (CCR) or accuracy, true positive rate (TPR) or sensitivity, true negative rate (TNR) or specificity, false positive rate (FPR), false negative rate (FNR), precision, recall, and F1 score. A formal definition of these performance metrics is shown in Table 7.

## 5. Experimental Design and Results

### 5.1. Experimental Design

A birth (term-preterm) dataset with 1300 patients' observations is obtained in order to perform the experiment. The experiment is carried out with the help of Python and Scikit-Learn library or under WEKA toolbox (http://www.cs.waikato.ac.nz/ml/weka). The observations in the birth dataset are carefully reviewed for prediction of birth cases. This is in fact a binary class dataset in which all births occurring between 28^th^ to 37^th^ weeks are termed as PTB class with label “1” whereas all births after 37^th^ weeks are termed as term birth (TB) class with label “0.” According to the study, around **24%** of the findings in the dataset are of PTB with label “1” and remaining **76%** are of TB with label “0.” Hence, PTB class is dominated by TB class, and we can say that PTB is the minority class and TB is the majority class. Therefore, there is a need of a good sampling technique for medical datasets [24, 52]. In this context, synthetic minority oversampling technique (SMOTE) is used to balance the target dataset [65]. This can be achieved by replicating the PTB cases until it reaches approximately 50% of the dataset. This gives a new balanced (term-preterm) dataset.

### 5.2. Results and Discussion

A total of 1300 patients (women) were selected in this study based on inclusion-exclusion criteria. Out of 1300 pregnant women, 309 women were having preterm birth and rest 991 women were having term birth. Thus, the incidence of PTB is 23.78% of total pregnant women. In this work, the performance of DT, LR, and SVM classifiers is evaluated in terms of accuracy, specificity, and sensitivity [66]. With these indicators, it is possible to compare the proposed model performance with three classifiers. Tables 8 and 9 present the performance metrics of classifiers for the original dataset and balanced dataset, respectively.

Based on the results shown in Tables 8 and 9, we can observe that the accuracy of three different classifiers is roughly around 85%. With respect to the original dataset, the accuracy of SVM is 86.1% which is highest, followed by LR and DT. The results were additionally improved (after applying SMOTE) with the balanced dataset. The accuracy of SVM classifier in the balance dataset increases from 86.1% to 90.9% compared with original dataset. In summary, the SVM model is the best classifier in the experiment.

## 6. Conclusion and Future Scope

In this study, the proposed model (RPCM) can be used for prediction of PTB based on excellent features (text-based symptoms) available in obstetrical data. The work focuses on feature selection (entropy-notion) approach by applying machine learning classifiers (DT, LR, and SVM) in order to classify all birth cases into term birth and PTB. Comparing the performances of the classifiers, it is evident that SVM classifier is the most suitable classifier as it achieves an accuracy of 90.9%. According to the findings of this study, the identified risk factors (excellent features) will be helpful in the prediction of PTB, especially in rural community. The developed model supports the decision-making process in maternity care by identifying and alerting the pregnant women at risk of preterm delivery thereby preventing possible complications, reducing the diagnosis cost, and ultimately minimizing the risk of PTB. The present system can be regarded as a successful innovation in Obstetrics to give clinical support to patients during pregnancy consultations. In particular, RPCM claims to assist healthcare professionals to make effective and timely decisions without consulting specialists directly.

The limitation of the present research is that the risk factors for PTB are limited in size and dataset is small, which could be increased to improve the performance of the PTB prediction in the future studies. However, expert knowledge and clinical judgement may still be needed to interpret this risk and take appropriate action in individual cases.

## Figures and Tables

**Figure 1:** Conceptual model for feature selection approach.

**Figure 2:** Framework of the proposed model.

**Figure 3:** A conceptual PTB prediction model.

**Table 1:** Definitions used in the present study.

Terminology	Description
Antenatal care	Antenatal care (ANC) refers to the fundamental, clinical, and nursing care suggested for ladies during pregnancy
Neonate	A neonate or a newborn infant is a child under 28 days of age
Neonatal death	A death during the first 28 days of life (0–27 days) is termed as a neonatal death
Live birth	A birth at which a child is born alive is termed as live birth
Term birth	A birth at the end of a normal duration of pregnancy between 37 and 40 weeks of gestation is termed as term birth
Maternal death	A maternal death is the death of a woman while pregnant or within 42 days of termination of pregnancy
Stillbirth	Stillbirth is the delivery, after the 20th week of pregnancy, of a baby who has died
Abortion	Termination of a pregnancy either medically or induced
Miscarriage	Natural loss of pregnancy during first trimester
Gestational age	Gestational age (GA) refers to the time from the first day of a woman's last menstrual period to birth

**Table 2:** Summary of the obstetrical (term-preterm) dataset.

Problem name	Number of features	Number of classes	Number of instances
Birth case	36	2	1300

**Table 3:** Maternal features associated with PTB.

S. no.	Feature ID	Feature name
1	PID	Patient identification
2	WA	Woman age
3	LMP	Last menstrual period
4	EDD	Estimated delivery date
5	G	Gravida
6	P	Parity
7	A	Abortion
8	L	Living
9	EL	Educational level
10	H	Height
11	W	Weight
12	BMI	Body mass index
13	BP	Blood pressure
14	HB	Hemoglobin
15	ANC	Antenatal care visit
16	ADD	Actual delivery date
17	OH	Obstetric history
18	PCS	Previous caesarean section
19	GA	Gestational age
20	BW	Birth weight
21	GDM	Gestational diabetes mellitus
22	FHR	Fetal heart rate
23	MG	Multiple gestation
24	ND	Normal delivery
25	MH	Previous medical history
26	LBW	Low birth weight
27	ASPX	Asphyxia
28	HT	Hypertension
29	PE	Preeclampsia
30	LV	Live birth
31	SB	Still birth
32	OB	Obesity
33	AN	Anemia
34	TH	Thyroid
35	NS	Neonatal status
36	PTB	Preterm birth

**Table 4:** Summary of discretized (term-preterm) dataset.

Outcome	*N*
Number of features	36
Number of classes	2
Total instances	1300
Term birth	991
Preterm birth	309

**Table 5:** List of excellent features in discretized (term-preterm) dataset.

Feature code	Feature name	Feature type
WA	Woman age	Numeric
PT	Parity	Numeric
GD	Gravida	Numeric
BMI	Body mass index	Ordinal
ANC	Antenatal care visit	Numeric
GA	Gestational age	Numeric
FHR	Fetal heart rate	Numeric
BP	Blood pressure	Ordinal
HB	Hemoglobin	Numeric
GDM	Gestational diabetes mellitus	Binary
PE	Preeclampsia	Binary
HT	Hypertension	Binary
OH	Obstetric history	Binary
EL	Education level	Ordinal
CS	Previous caesarean section	Binary
MH	Previous medical history	Binary
PTB	Preterm birth (target variable)	Binary

**Table 6:** Confusion matrix.

	Predictive positive	Predictive negative
Actual positive	True Positive (TP)	False Negative (FN)
Actual negative	False Positive (FP)	True Negative (TN)

**Table 7:** Performance metrics for machine learning classifiers.

Metrics	Formula
CCR	((TP+TN)/(TP+FP+FN+TN))%
TPR	TP/(TP+FN)
TNR	TN/(TN+FP)
FPR	FP/(TN+FP)
FNR	FN/(TP+FN)
Precision	TP/(TP+FP)
Recall	TP/(TN+FN)
*F*_1_ score	2*∗*TP/(2*∗*TP+Fp+FN)

**Table 8:** Performance metrics of the classifiers—original dataset.

Classifiers	Accuracy	Sensitivity	Specificity
DT	0.777	0.702	0.930
LR	0.841	0.863	0.971
SVM	**0.861**	0.801	0.702

**Table 9:** Performance metrics of the classifiers—balanced dataset.

Classifiers	Accuracy	Sensitivity	Specificity
DT	0.796	0.713	0.972
LR	0.872	0.832	0.954
SVM	**0.909**	0.891	0.783

## Data Availability

The data used to support the finding of this study are available from the corresponding author upon reasonable request. The data are not publicly available due to privacy and ethical restrictions of Institutional Ethics Committee.
